This article has been retracted.

# International Trade Path with Multi-Polarization based on Multidirectional Mutation Genetic Algorithm Enabled Neural Network

**DOI:** 10.1155/2021/1370180

**Published:** 2021-10-14

**Authors:** Qing Zhang, Choo Wei Chong, Abdul Rashid Abdullah, Mass Hareeza Ali

**Affiliations:** School of Business and Economics University Putra Malaysia, Serdang, Selangor Darul Ehsan 43400, Malaysia

## Abstract

At present, the development speed of international trade cannot catch up with the economic development speed, and the insufficient development speed of international trade will directly affect the rapid development of national economy. In order to solve the problem of international trade, the overall optimal scheduling of trade vehicles and the optimal planning of trade transportation path are very important to improve enterprise services, reduce enterprise costs, increase enterprise benefits, and enhance enterprise competitiveness. The second development of the program is based on the programming interface provided by Baidu map. This paper proposes a neural network algorithm for genetic optimization of multiple mutations, which overcomes the shortcoming of traditional genetic algorithm population “ten” character distribution by mixing multiple coding methods, and enhances the local search ability of genetic algorithm by introducing a new large-mutation small-range search population. The example application shows that the optimization method can realize the optimization of international trade path under real road conditions and greatly improve the work efficiency of actual trade.

## 1. Introduction

The development speed of international trade cannot keep up with the economic development speed. Traditional trade is based on the use of paper map or experience to make trade plans manually. The goods transported are often in small batches and in large quantities. To a certain extent, the low level of trade hinders the rapid development of the national economy, resulting in idleness of vehicles, low floor area ratio of freight cars, and high-speed transportation of goods. Due to the low operation efficiency of the trade system, such as vehicles traveling to and from repeated road sections, the timeliness of traditional trade is poor, and the trade cost is high, which makes it difficult to meet the high service requirements of customers. It also increases the burden of urban traffic and has a negative impact on traffic and environment.

For the study of path optimization, Yang et al. studied a dynamic optimization problem, in which the vehicle speed varies with time and region [1]. In this paper, the traffic time of urban road network is predicted by Fu and Smith. The traffic time of morning peak, evening peak, and normal urban road is predicted by using neural network, and the actual data is used for testing [2]. Soumia et al. obtained the driving time of the vehicle by using the vehicle speed and the distance between the points expressed by the time-varying function [3]. Martin put forward a travel time function model, which pushed back the starting time by arrival time, and verified it with actual traffic data [4]. Zhang and Huang studied the dynamic route selection problem of urban logistics and studied the selection model by using the road data collected by floating cars [5]. Wang et al. considered the characteristics of vehicle speed changing with time and road section in real road network and simulated the road speed in different time periods for analysis close to the actual situation [6]. Shi et al. studied the application of Baidu map API in vehicle routing problem and obtained the actual path between two points through Baidu map API [7]. But the traditional mathematical methods such as linear programming cannot get satisfactory results.

This paper is divided into five parts. The first part is the background. The second part is the literature review, analysis of the research results. The third part is the introduction of optimization and neural network algorithm based on multidirectional mutation genetic optimization. The fourth part is the specific experimental analysis, showing the realization of trade path optimization based on multidirectional mutation genetic optimization neural network algorithm. The fifth part is the conclusion.

## 2. Related Work

In real life, many aspects are related to problems, such as path planning, network optimization, and economic investment. There are optimization problems in almost all areas of the real world. It has always been the focus of scholars. At present, optimization algorithms are mainly divided into traditional accurate algorithms and intelligent optimization algorithms. Since the complexity of traditional accurate algorithms increases exponentially with the expansion of the scale of the problem, the focus of scholars has gradually turned to intelligent optimization algorithms since the 1980s. Zhang et al. proposed simulated annealing algorithm (SA) to simulate the annealing process of metals and successfully applied it to solve TSP [8]. Hirschfeld et al. proposed a fine-tuned Lin–Kernighan algorithm, which can well solve the optimization problem [9]. In recent years, Seeland and Mäder proposed a hybrid multi-particle swarm optimization algorithm to study the probability-based traveling salesman problem [10]. Zhou et al. proposed a hybrid multidirectional mutation algorithm by combining local optimization with generalized segmentation crossover operator, which improved the efficiency of the algorithm to a certain extent [11]. Farrell et al. improved the crossover operation of multidirectional mutation algorithm and designed a sequential crossover operator to improve the quality of the optimal solution [12]. Chen et al. combine the greedy algorithm with the mutation operation of multidirectional mutation algorithm to design a new greedy mutation operator to improve the efficiency of multidirectional mutation algorithm in solving optimization problems [13].

Goh et al. used the dynamic programming method to solve the optimization of fixed number of vehicles [14]. Huang et al. studied the dynamic optimization, applied it to medicine distribution, and finally got a better solution [15]. Abbas et al. studied the optimization of multiple distribution points with time window constraints based on multidirectional mutation algorithm [16]. By combining the TABU list characteristics of simulated annealing method and TABU search method, Zhong et al. solved the optimization problem, and the result was better than that of single simulated annealing algorithm [17]. Jouppi et al. divided the optimization process into two stages: first simplifying the optimization to TSP and then solving TSP. This is a relatively new method and achieved good results [18]. Huang et al. proposed a new path merging method and path length saving value calculation formula, improved the classical saving method to solve the optimization, and improved the performance of the original algorithm [19]. Deng et al. studied the optimization of multi-cycle and multi-distribution center [20]. Liu et al. studied the optimization of random demand of distribution points and proposed a two-stage simulated annealing algorithm to solve it [21]. Ghorbani et al. improved the selection operator and cross mutation rate of the multidirectional mutation algorithm [22]. Qiao et al. used multi-directional mutation algorithm to simulate the minimum cost model based on the technology of traffic flow [23]. Kim et al. studied a kind of distribution problem under the condition of full load [24]. It can be seen from the results that the traditional mathematical methods such as linear programming cannot get satisfactory results. In recent decades, with the rapid development of computational intelligence, some intelligent optimization algorithms, which are completely different from the classical mathematical programming principles, have appeared. Genetic algorithm (GA) has been well received by the academia for its excellent global search ability, implicit parallelism, and simple operators, and it has become one of the hot technologies to solve optimization problems in recent years.

## 3. Construction of Optimization Model Based on Multidirectional Mutation Genetic Algorithm Enabled Neural Network

### 3.1. Brief Introduction of Path Optimization Model

Path optimization is a mathematical problem. It is a classical problem in graph theory and a typical combinatorial optimization problem. The problem is described as follows: a businessman wants to travel to *n* cities to sell goods, and he knows the distance between any two cities. Starting from city *X*, he needs to find a route that passes through all cities once and only once, and finally returns to city *X* to minimize the total distance. As shown in Figure 1, the traveling salesman problem of 100 cities is solved. Optimization seems to be a relatively simple problem, but its description is simple and it is easy to understand. However, the complexity of its solution increases exponentially with the scale of the problem, which is difficult to solve by traditional algorithms.

The following model can be established. Set *n* points, and *i* ∈ *V*, respectively, number 1,2,…, *n*, given a completely undirected graph *G*=(*V*, *E*), *C*={1,2,…, *n*}, *n* > 1 where each point, each side (*i*, *j*) ∈ *E* has a non-negative integer consumption *D*_*i*,*j*_, *ij* ∈ *V*, and formula (1):

(1) $$\begin{array}{c} X_{i,j}=\left\{\begin{array}{cc} 1, & \text{edge}\left(i,j\right)\text{ is on the optimal route},\\ 0, & \text{others.} \end{array}\right. \end{array}$$

A feasible path of *G* is to pass every vertex of *V* exactly once, and the consumption is the weight of all edges and *W*. Therefore, the optimization problem is to find out the circuit with minimum *G* in *W*.

(2) $$\begin{array}{c} W=\sum D_{i,j}X_{i,j}, \end{array}$$

(3) $$\begin{array}{c} \sum_{j=1}x_{i,j}=1,\;i\in V, \end{array}$$

(4) $$\begin{array}{c} \sum_{i=1}x_{i,j}=1,\;j\in V, \end{array}$$

(5) $$\begin{array}{c} \sum_{i,j\in S}x_{i,j}\leq \left|S\right|-1,\;S\subseteq V,2\leq \left|S\right|\leq n-2. \end{array}$$

(6) $$\begin{array}{c} x_{i,j}\in \left\{0,1\right\},\;i,j\in V,i\neq j, \end{array}$$

where |*S*| is the number of vertices. Equation (2) is the objective function, which requires the minimum objective function. Expressions (3) and (4) denote passing through each vertex once and only once; that is, each vertex has only one edge in and one edge out. Equation (5) guarantees that there is no sub-loop solution. The values of *i* and *j* are given by formula (6).

International trade route selection refers to the fact that there are a certain number of customers who trade goods from the trade center to these customers who have a certain demand for goods. There are a number of vehicles in charge of trade. These vehicles are dispatched, and the appropriate driving route is planned to meet the customers' demand for goods. Vehicle routing problem in trade is a famous NP hard problem in combinatorial optimization. Since optimization was put forward in 1959, it has been one of the basic problems of optimization and has attracted the attention of experts and scholars. Because optimization is widely used and of great significance for economic and social development, the research on optimization has never stopped at home and abroad. Optimization can be described as shown in Figure 2.

#### 3.1.1. The Elements Included in Optimization

*(1) Road*. It is the optimal infrastructure and basic conditions, which is one of the core elements. Road is the basis of goods transportation and one of the core elements of optimization. The generated optimal (near optimal) path is usually based on the basic characteristics of the road network (such as road condition, distance, connectivity, etc.) and returns to the trade center from the trade center unless passing through customers in turn.

*(2) Customer*. It (such as demand stores) represents the service objects, which usually include demand goods types, demand service time, demand uncertainty, and demand priority.

*(3) Trade Centre*. The start or end of each vehicle. Vehicles trade goods with customers from the trade center. In practice, after the goods trade, the vehicles return to the trade center.

*(4) Vehicles*. To complete the trade activities from the trade center to the customers, we need certain vehicles. Compared with vehicles for other purposes, vehicles for trade generally include the place of departure and return of the vehicle (whether to return to the trade center after completing the task), the limit of load and volume of the vehicle, and the cost of using the vehicle.

*(5) Transportation Arrangement Requirements*. In the process of trade, vehicle routes often need to meet the relevant needs of customers and vehicle restrictions, according to the needs and conditions of transportation arrangements, such as vehicle trade goods that cannot exceed the vehicle's carrying capacity, and in the time required by customers, etc.

To sum up, the goal of optimization is usually considered from the following aspects: the minimum total running time, the minimum total transportation cost, the minimum total transportation distance, the minimum number of vehicles required to complete the task, the minimum penalty value of service not completed according to the specified requirements, etc.

Construction of optimization model based on multidirectional mutation genetic algorithm enabled neural network. Intelligent optimization algorithm has global optimization performance, strong versatility and is suitable for parallel processing [25–28]. It can effectively solve some complex optimization problems. This paper proposes a neural network algorithm for genetic optimization of multiple mutations, which overcomes the shortcoming of traditional genetic algorithm population “ten” character distribution by mixing multiple coding methods, and enhances the local search ability of genetic algorithm by introducing a new large mutation small range search population. (1) A coding structure is used to transform the solution into a genetic code satisfying the constraint conditions, which is similar to the chromosome structure and is convenient for genetic operation. It is usually represented by bit string or string. (2) Using random method to generate individuals as the initial population, the size of the general population needs to be set larger. It shows that population diversity can better complete the inheritance of excellent genes. (3) The design of fitness function: fitness function is mainly used to express the advantages and disadvantages of individuals, distinguish the advantages and disadvantages of individuals, as the basis of multidirectional mutation algorithm, and also represents the adaptability of individuals in the environment. (4) The design of selection operator: according to the fitness function designed in the previous step, the values are arranged from high to low. The higher the value is, the higher the probability of being selected is. Therefore, the next generation is generally the chromosome with high fitness. (5) The design of crossover operator: randomly select a pair of parent individuals, and generate two random numbers *P*1 and *P*2 between 0 and 1. If *P*1 < crossover probability Pc, two parents are crossed to generate new offspring. (6) The design of mutation operator: mutation is an indispensable link to imitate the chromosome mutation in nature. If *P*2 < mutation probability Pm, mutation operation was carried out for new offspring selection. (7) In the design of termination conditions, when the individual with the highest fitness in the population has not improved for several generations, or a certain number of iterations can be set to terminate. When convergence is not reached, go to step (1); otherwise, proceed to the next step. (8) The individual with the best fitness value in the output population: the flowchart of genetic optimization neural network based on multi direction mutation is shown in Figure 3.

### 3.2. Analysis of Path Optimization in Multilevel Trade

The trade destination (the first level is the trade site; the second level is the community level customer point) is often not scale level in real life and needs the best route optimization. Therefore, this paper attempts to use the dynamic programming method to solve the trade problem under the optimization model.

Dynamic programming is a method for solving multistage decision-making problems. The solution is to transform a multistage problem into a sub-stage problem with a certain recurrence relation, which simplifies the calculation process to a certain extent. The advantage of dynamic programming method is that it can get the optimal solution in a short time when the number of destinations is small. Its disadvantage is that with the increase of the number of destinations, it needs to save the value in the process of operation and consumes a lot of memory space, which restricts the dynamic programming method to solve the scale traveling salesman problem.

The dynamic programming method obtains the optimal solution of each sub-problem from the bottom up, so as to get the optimal solution of the final problem step by step. The dynamic programming method is divided into three steps according to the process: the first step transforms the initial problem into multiple interrelated sub-problems; the second step analyses this problem. Whether it meets the optimality principle and finds out the correct recursive relationship, the third step uses the recursive relationship to calculate upward to realize dynamic programming and obtain the results. In the optimization solution, the specific process is as follows: assuming that the trade center is 0 and needs to trade for customers 1, 2, and 3, the distance between each two points is shown in Figure 4; then the shortest distance is shown in equation (7), where *C*_*i*,*j*_ represents the distance from *i* to *j*.

(7) $$\begin{array}{c} d\left(0,\left\{1,2,3\right\}\right)=\min\left\{C01+d\left(1,\left\{2,3\right\}\right),C02+d\left(2,\left\{1,3\right\}\right),C03+d\left(3,\left\{1,2\right\}\right)\right\}. \end{array}$$

This is the final stage of decision-making, which must be based on the calculation results of *d*(1, {2,3}, *d*(2, {1,3})) and *d*(3, {1,2}), as shown in the following equations:

(8) $$\begin{array}{c} d\left(1,\left\{2,3\right\}\right)=\min\left\{C12+d\left(2,\left\{3\right\}\right),C13+d\left(3,\left\{2\right\}\right)\right\}, \end{array}$$

(9) $$\begin{array}{c} d\left(2,\left\{1,3\right\}\right)=\min\left\{C21+d\left(1,\left\{3\right\}\right),C23+d\left(3,\left\{1\right\}\right)\right\}, \end{array}$$

(10) $$\begin{array}{c} d\left(3,\left\{1,2\right\}\right)=\min\left\{C31+d\left(1,\left\{2\right\}\right),C32+d\left(2,\left\{1\right\}\right)\right\}. \end{array}$$

One more step from bottom to top can be expressed as below:

(11) $$\begin{array}{c} d\left(1,\left\{2\right\}\right)=C12+d\left(2,\left\{\right\}\right),\\ d\left(2,\left\{3\right\}\right)=C23+d\left(3,\left\{\right\}\right),\\ d\left(3,\left\{2\right\}\right)=C32+d\left(2,\left\{\right\}\right), \end{array}$$

(12) $$\begin{array}{c} d\left(1,\left\{3\right\}\right)=C13+d\left(3,\left\{\right\}\right),\\ d\left(2,\left\{1\right\}\right)=C21+d\left(1,\left\{\right\}\right),\\ d\left(3,\left\{1\right\}\right)=C31+d\left(1,\left\{\right\}\right). \end{array}$$

The specific calculation diagram is shown in Figure 5.

## 4. Empirical Analysis

### 4.1. Optimal Realization of Multidirectional Mutation Genetic Optimization Neural Network Algorithm

In this paper, a neural network algorithm for multiple mutation genetic optimization is first designed, and the parameters are set as follows: the population size is 100, the crossover probability Pc is 0.9, the mutation probability (1 − 0.9)*∗*Pm, where Pm is 0.9, and the evolution algebra is 400. Run 500 times. Because the objective function of the first level is the shortest total time, we focus on the final trade time. The number of runs and the optimal trade time obtained each time, as well as the algebraic corresponding graph of its occurrence, are shown in Figures 6 and 7.

Through the design of neural network algorithm optimized by multiple mutation genetics, there is nearly 60% probability to get the actual optimal solution (14449), and there is nearly 40% probability to get the suboptimal solution (15087), and the suboptimal solution is only 4.4% larger than the optimal solution, which is an acceptable satisfactory solution. The algebra of the optimal solution is mostly concentrated in 50–200 generations, which shows that the convergence speed of the genetic algorithm is also relatively satisfactory.

Similarly, neural network algorithm for genetic optimization of multiple mutations in the second layer runs 500 times. Because the objective function of the second level is the shortest total distance, we focus on the final trade distance. The number of runs and the optimal trade distance obtained each time, as well as its algebraic corresponding graph, are shown in Figures 8 and 9.

### 4.2. Implementation of Trade Route Optimization Algorithm Based on Multidirectional Mutation Genetic Algorithm Enabled Neural Network Algorithm

Based on the multidirectional mutation genetic optimization neural network algorithm, the improved multidirectional mutation algorithm is superior to the original genetic algorithm in solving results, iterations, and stability. Compared with the optimal result of genetic algorithm, the optimal result is reduced by 10.14% on average, and the average algebra of the optimal solution is smaller, which indicates that the convergence speed is faster. In addition, the volatility of the solution is much better than genetic algorithm, which has obvious advantages. The distribution diagram of the optimal solution of 100 runs is shown in Figure 10. The abscissa represents the number of runs, and the ordinate represents the total time of distribution.

The comparison diagram of the evolutionary convergence process of the multidirectional mutation genetic algorithm enabled neural network algorithm, and the genetic algorithm is shown in Figure 11. The abscissa represents the evolutionary algebra, and the ordinate represents the optimal value of the objective function in the population. In this case, it is the shortest total delivery time. It can be seen from the figure that the quality of the initial population of the multidirectional mutation genetic optimization neural network algorithm is obviously better than that of the genetic algorithm, and the convergence speed of the multidirectional mutation genetic optimization neural network algorithm is faster. And the final optimal solution is also better than that of the genetic algorithm.

Comparing the results of genetic algorithm and multidirectional mutation genetic optimization neural network algorithm, it can be found that due to the improvement of the mutation operator, the results of multidirectional mutation genetic optimization neural network algorithm have less path crossing, while the results of genetic algorithm have more path crossing. Therefore, from the point of view of the shortest time of distribution and the total distance of driving, the results of IgA are better than those of GA.

In order to better observe the effect of each improvement mode, two modes are set in this section: only improving the initial population, only improving the mutation operator and adaptive adjusting the cross mutation rate. Combining the results of genetic algorithm and multidirectional mutation genetic optimization neural network algorithm, the traffic data at 11 : 00 noon on a Sunday is used, and the results are shown in Figure 12.

The blue line represents the evolutionary convergence process of genetic algorithm. The purple line represents the genetic algorithm, which only improves the mutation operator and adaptively adjusts the crossover mutation rate. It can be seen that the convergence speed of the improved genetic algorithm is obviously faster, and it can jump out of the local optimal situation, and the final result is better than that of the genetic algorithm. The green line indicates the genetic algorithm which only improves the initial population generation. It can be seen that the quality of the initial population of the improved genetic algorithm is already very high, and the value of the objective function is far less than that of the genetic algorithm, which randomly generates the initial population. It can be seen that the evolution of green line is very little in the later stage. The red line indicates the evolutionary convergence process of the multidirectional mutation genetic optimization neural network algorithm. It can be seen that the multidirectional mutation genetic optimization neural network algorithm combines the advantages of the purple line and the green line, which not only has high quality of the initial population, but also is easy to jump out of the local optimum.

To sum up, the genetic optimization neural network algorithm based on multidirectional mutation improves the quality of the initial population and speeds up the optimization speed through the improvement of the generation mode of the initial population. Through the improvement of the mutation operator, it improves the goodness of solution and the diversity of the population. Through the adaptive adjustment of the crossover rate and mutation rate, it is conducive to jump out of the local optimum and improve the convergence speed.

## 5. Conclusion

Based on the analysis of references, this paper focuses on the trade route optimization under real road conditions. The work and conclusions of this paper are as follows: the classification of trade is studied. According to the actual situation, trade is divided into “trade” and “bulk goods trade” with different characteristics. The “trade” is divided into two levels according to the actual situation. The first level is from the distribution center of the destination to the trade station. The second level is the transportation personnel from the trade site to trade to customers. These two levels have different characteristics and application requirements. This paper studies the trade path planning problem, analyses the TSP, optimization model, theory and algorithm, and concludes that the international trade in the real situation has a high similarity with optimization, and the international trade of bulk goods has a high similarity with optimization, so the practical problems can be connected with the theoretical model. The example shows that the quality of the initial population is improved, and the optimization speed is accelerated by the improvement of the generation mode of the initial population. The excellent degree of the solution and the diversity of the population are improved by the improvement of the mutation operator. The adaptive adjustment of the crossover rate and the mutation rate is conducive to jump out of the local optimum and improve the convergence speed. The improved neural network algorithm based on multidirectional mutation genetic optimization has some advantages.

## Figures and Tables

**Figure 1:** Traveling salesman problem in 100 cities.

**Figure 2:** Vehicle routing problem.

**Figure 3:** Flowchart of multidirectional mutation genetic optimization neural network algorithm.

**Figure 4:** The distance between points.

**Figure 5:** Dynamic programming method to solve optimization flowchart.

**Figure 6:** The first-level optimal solution at 15 : 00 on Tuesday.

**Figure 7:** The algebra where the first-level optimal solution appears at 15 : 00 on Tuesday.

**Figure 8:** The second-level optimal solution at 15 : 30 on Tuesday.

**Figure 9:** The algebra where the second-level optimal solution appears at 15 : 30 on Tuesday.

**Figure 10:** The optimal solution distribution for 100 runs.

**Figure 11:** Comparison of evolutionary convergence process.

**Figure 12:** Comparison diagram of evolutionary convergence process.

## Data Availability

The data used to support the findings of this study are available from the corresponding author upon request.
